The article "Id-1 stimulates cell proliferation through activation of EGFR in ovarian cancer cells" was retracted in 2021. Reasons: duplicated images; concerns about the data.

# Id-1 stimulates cell proliferation through activation of EGFR in ovarian cancer cells

**DOI:** 10.1038/sj.bjc.6602254

**Published:** 2004-12-14

**Authors:** X Zhang, M-T Ling, H Feng, Y C Wong, S W Tsao, X Wang

**Affiliations:** 1 Cancer Biology Group, Department of Anatomy, The University of Hong Kong, 1/F, Faculty of Medicine Building, 21 Sassoon Road, Hong Kong

**Keywords:** Id-1, EGFR, cell proliferation, ovarian cancer

## Abstract

Increased EGFR (epidermal growth factor receptor) expression has been reported in many types of human cancer and its levels are positively associated with advanced cancers. Recently, upregulation of Id-1 (inhibitor of differentiation or DNA binding) protein was found in over 70% of ovarian cancer samples and correlated with poor survival of ovarian cancer patients. However, the molecular mechanisms responsible for the role of Id-1 in ovarian cancer are not clear. The aim of this study was to investigate the effect of Id-1 on ovarian cancer proliferation and its association with the EGFR pathway. To achieve this, we transfected an Id-1 expression vector into three ovarian cancer cell lines and examined cell proliferation rate by flow cytometry and bromodeoxyuridine staining. We found that ectopic Id-1 expression led to increased cell proliferation demonstrated by increased BrdU incorporation rate and S-phase fraction. The Id-1-induced cell growth was associated with upregulation of EGFR at both transcriptional and protein levels. In contrast, inactivation of Id-1 through transfection of an Id-1 antisense vector resulted in downregulation of EGFR. Our results indicate that increased Id-1 in ovarian cancer cells may promote cancer cell proliferation through upregulation of EGFR. Our findings also implicate that Id-1 may be a potential target for the development of novel strategies in the treatment of ovarian cancer.

Ovarian cancer is the second leading cause of death from gynaecologic malignancy worldwide, with a mortality rate of 114.2 per 100 000 women (Parkin *et al*, 2001). Approximately 75% of women present with ovarian cancer at advanced stage; therefore, prognosis for this disease is poor, with a 5-year survival rate of less than 40% (Jemal *et al*, 2004).

Although the molecular basis for the development of ovarian cancer is not clear, upregulation of the epidermal growth factor receptor (EGFR) is reported to be a frequent event in ovarian cancer and associated with tumour progression, invasion and poor survival rate (Kohler *et al*, 1989; Simpson *et al*, 1995; Skirnisdottir *et al*, 2001; Cloven *et al*, 2004). For example, expression of EGFR is significantly higher in malignant ovarian cancer cells compared to borderline and benign tumours (Simpson *et al*, 1995). A study on 226 patients with different stages of ovarian cancer found that EGFR-positive staining was evident in approximately 50% of the patients, and among them 59.8% had recurrent or died of this disease (Skirnisdottir *et al*, 2004). Furthermore, in a separate study, the survival time of patients (*n*=111) with EGFR-positive tumour was much shorter than patients with EGFR-negative tumours (Kohler *et al*, 1989). These results indicate that EGFR may be a key factor in promoting ovarian cancer growth as well as progression. Recently, using antisense technology, suppression of EGFR led to inhibition of cellular proliferation, cell adhesion and tumorigenicity in ovarian cancer cells (Alper *et al*, 2000). In addition, targeting the EGFR using an active EGFR-specific tyrosine kinase inhibitor ZD1839 also resulted in the reduction of ovarian cancer cell growth (Sewell *et al*, 2002). These results further suggest that inactivation of EGFR pathway may provide a therapeutic target for the treatment of ovarian cancer. However, the molecular basis of the EGFR-induced ovarian cancer cell proliferation is still not clear.

The article "Id-1 stimulates cell proliferation through activation of EGFR in ovarian cancer cells" was retracted in 2021. Reasons: duplicated images; concerns about the data.

Recently, Id-1 (inhibitor of differentiation or DNA binding) has been suggested as one of the upstream regulators of the EGFR pathway (Ling *et al*, 2004). Id-1 is a member of the helix–loop–helix (HLH) transcription factor family. It lacks the basic domain for DNA binding and acts as a dominant inhibitor of the basic HLH transcription factors by forming heterodimers (Benezra *et al*, 1990). Like EGFR, upregulation of Id-1 is frequently found in many types of human cancer such as breast (Lin *et al*, 2000), pancreas (Maruyama *et al*, 1999), cervical (Schindl *et al*, 2001), head and neck (Langlands *et al*, 2000) and prostate cancer (Ouyang *et al*, 2002a), and increased Id-1 expression levels are associated with advanced tumour stage and poor prognosis (Maruyama *et al*, 1999; Schindl *et al*, 2001; Ouyang *et al*, 2002a). Recently, it is reported that over 70% of ovarian cancer samples (among a total of 101 cases) are found to express Id-1 protein, while none of the nonmalignant cystadenomas shows positive Id-1 staining examined by immunohistochemistry as well as Western blotting (Schindl *et al*, 2003). In addition, the cancer samples with poor or moderate histological differentiation show stronger Id-1 expression than the well-differentiated tumours. Furthermore, the overall survival is much shorter in the patients with higher Id-1 expression than the patient with relatively lower Id-1 expression (Schindl *et al*, 2003). These results indicate that Id-1 may play an important part not only in tumorigenesis but also progression of ovarian cancer.

The article "Id-1 stimulates cell proliferation through activation of EGFR in ovarian cancer cells" was retracted in 2021. Reasons: duplicated images; concerns about the data.

The fact that both Id-1 and EGFR protein expression levels increase with progression and poor prognosis as well as chemoresistance of ovarian cancer (Alper *et al*, 2001; Maihle *et al*, 2002; Schindl *et al*, 2003; Cloven *et al*, 2004) raises a hypothesis that these two proteins may either share similar functions or regulate through same pathways. In addition, evidence from our previous studies has shown that Id-1 promotes prostate cancer cell proliferation through activation of EGFR (Ling *et al*, 2004), indicating that Id-1 may be an upstream regulator of EGFR. To study the role of Id-1 on ovarian cancer cell growth and its association with EGFR pathway, in this study, we first transfected an Id-1 expression vector into three ovarian cancer cell lines and then examined the effect of ectopic Id-1 expression on ovarian cancer cell proliferation using bromodeoxyuridine (BrdU) staining and flow cytometric analysis. The effect of Id-1 on EGFR expression at both transcriptional and protein levels was also determined by luciferase assay and Western blotting. These results were further verified through transfection of an antisense Id-1 vector in two ovarian cancer cell lines with high levels of Id-1. Our results suggest that ectopic Id-1 expression stimulates ovarian cancer cell proliferation and this process is mediated through upregulation of EGFR. Our results provide novel evidence to suggest Id-1 as an upstream regulator of the EGFR pathway in promoting ovarian cancer cell growth.

## MATERIALS AND METHODS

### Cell lines and cell culture conditions

Five ovarian cancer cell lines, Skov3 (obtained from ATCC, Manassas, VA, USA), Ovca420, Ovca432, Ovca433, Ovca429, were maintained in RPMI 1640 (Life Technologies Inc., Carlsbad, CA, USA) supplemented with 2 mM L-glutamine and 5% (v v^−1^) foetal calf serum (FCS) at 37°C. Ovca420, Ovca432, Ovca433 and Ovca429 were established from freshly isolated ascites or tumour explants from patients with late-stage ovarian adenocarcinomas with distinct characteristics (Rauh-Adelmann *et al*, 2000).

### Generation of stable Id-1-expressing transfectants

The pBabe–Id-1 retroviral expression vector and its corresponding vector control were used for generation of stable transfectants. Details on the vectors as well as transfection procedures have been described previously (Ouyang *et al*, 2002b). All the transfectants were selected and maintained in puromycin (1–2 *μ*g ml^−1^). The pool of more than 20 individual clones transfected with either Id-1 or pBabe was generated. Cell culture medium was changed to serum-free medium (SFM) before performing additional experiments.

The article "Id-1 stimulates cell proliferation through activation of EGFR in ovarian cancer cells" was retracted in 2021. Reasons: duplicated images; concerns about the data.

### BrdU staining

Detailed experimental procedures have been described previously (Wang *et al*, 2002a). Briefly, monolayer **c**ells were grown on 4-mm Chamber slides (ICN, Biomedicals, Aurora, OH, USA) and the culture medium was changed to SFM for 48 h. Then, the cells were treated with BrdU (10 mM) for 1 h and then washed once with PBS. The cells were then fixed in cold methanol for 5 min at room temperature and washed in PBS. The cells were incubated with mouse monoclonal antibody against BrdU (1 : 10, Roche Diagnostics, Indianapolis, IN, USA) for 1 h at 37°C and then with anti-mouse IgG-FITC for 1 h at 37°C after washing with PBS. The percentage of FITC-positive cells was evaluated and at least 500 cells were evaluated in each experiment. The percentage of BrdU-positive cells in the control vector (pBabe) was considered as 100. The error bars represent the standard deviation generated from three independent experiments.

### Cell cycle analysis

Cells (5 × 10^5^) were plated in 5% FCS culture medium. After 24 h, the culture medium was replaced by SFM for 48 h. The cells were harvested by trypsinisation and then fixed in ice-cold 70% ethanol. The cells were then washed with PBS and incubated with propidium iodide (50 *μ*g ml^−1^) and RNase (1 *μ*g ml^−1^) for 30 min. Flow cytometric analysis was performed on an EPICS profile analyzer and analysed using the ModFit LT2.0 software (Coulter) as described previously (Wang *et al*, 2002a).

### Western blotting

Detailed experimental procedures were described previously (Ouyang *et al*, 2002b). Briefly, whole-cell lysate was prepared by resuspending cell pellet in lysis buffer (50 mM Tris-HCl (pH 8.0), 150 mM NaCl, 1% NP40, 0.5% deoxycholic acid, 0.1% SDS) including protease inhibitors (1 *μ*g ml^−1^ aprotinin, 1 *μ*g ml^−1^ leupeptin, 1 mM PMSF), and protein concentrations were measured using the protein assay kit (Bio-Rad, Hercules, CA, USA). Protein suspension from the whole-cell lysate (20 *μ*g) was loaded onto a sodium dodecylsulphate–polyacrylamide gel (SDS–PAGE) for electrophoresis and then transferred to a PVDF membrane (Amersham, Piscataway, NJ, USA). The membrane was then incubated with primary antibody for 1 h at room temperature against Id-1, EGFR, *β*-actin (Santa Cruz Biotechnology, Santa Cruz, CA, USA). After washing with TBS-T, the membrane was incubated with secondary antibody against mouse or rabbit IgG and the signals were visualised using ECL plus Western blotting system (Amersham, Piscataway, NJ, USA).

### Luciferase assay

Cells were plated into a 12-well plate at a density of 1 × 10^5^ cells well^−1^. After 24 h, the medium was changed to SFM. pER-1 (luciferase reporter containing the EGFR promoter, kindly provided by Dr A Johnson, NCI, MD, USA) and pRL-CMV-Luc (internal control) were cotransfected with either the pcDNA, pcDNA-Id-1 or pcDNA-Id-1-AS, respectively (Ling *et al*, 2004), into the cells using Fugene 6 reagent (Roche Diagnostics, Indianapolis, IN, USA). Cells were lysed 48 h after transfection and were assayed for luciferase activity using the Dual-luciferase reporter assay system (Promega, WI, USA). Each data point represented the mean of three experiments and error bars indicated the standard deviation.

The article "Id-1 stimulates cell proliferation through activation of EGFR in ovarian cancer cells" was retracted in 2021. Reasons: duplicated images; concerns about the data.

## RESULTS

### Generation of stable Id-1 transfectants in ovarian cancer cells

Under *in vitro* culture conditions, Id-1 expression is usually dependent on FCS stimulation and this characteristic is more evident in cell lines exhibiting less aggressive phenotype. For example, the androgen- or oestrogen-dependent cell lines (i.e. LNCaP (prostate cancer) and MCF7 (breast cancer)), which represent less aggressive tumours, show serum-dependent Id-1 expression. In contrast, the androgen- or oestrogen-independent cell lines (i.e. PC3 (prostate cancer) and MDA-MB-231 (breast cancer)), which represent aggressive tumours, express the Id-1 protein constitutively regardless of serum concentrations (Lin *et al*, 2000; Ouyang *et al*, 2002b). This phenotype provides a tool for studying the direct role of Id-1 on human cancer cells through either ectopic introduction or inactivation of the Id-1 gene. In this study, we first examined Id-1 protein expression in five ovarian cancer cell lines in a range of FCS concentrations (5, 2.5, 1 and 0%). As shown in Figure 1A

**Figure 1:** Effect of FCS on Id-1 expression in ovarian cancer cell lines and Id-1 expression in stable transfectants. (**A**) Western blotting analysis of Id-1 protein expression in five ovarian cancer cell lines, Ovca420, Ovca432, Ovca433, Ovca429 and Skov3, in culture medium containing different serum concentrations. Note that the expression of Id-1 is dependent on FCS in Ovca420, Ovca432 and Ovca433 cell lines but independent in Ovca429 and Skov3 cell lines. (**B**) Three cell lines Ovca420, Ovca432 and Ovca433 were transfected with an Id-1 expression vector (pBabe–Id-1) or the empty control (pBabe) and stable transfectants were generated. Id-1 protein expression was examined by Western blotting after culturing in SFM for 48 h. Expression of actin was examined as an internal loading control. Note that Id-1 protein levels are much higher after ectopic expression of the pBabe–Id-1 vector in Ovca420, Ovca432 and Ovca433 cell lines. Results represent three experiments.

, ovarian cancer cell lines Ovca420, Ovca432 and Ovca433 showed a serum-dependent Id-1 expression, while the expression of Id-1 was much less serum dependent in the Ovca429 and Skov3 cells. The Id-1 expression pattern in these ovarian cancer cell lines also seemed to correlate with their malignant phenotype. For example, Ovca429 cell line has been reported to be much more aggressive demonstrated by its highly invasive nature and increased expression of metastasis promoting proteins such as uPA and MMP compared to Ovca432 and Ovca432 cells (Ellerbroek *et al*, 1998; Ahmed *et al*, 2002). We then transfected an Id-1 expression vector into Ovca420, Ovca432 and Ovca433 cell lines and generated stable transfectants. As shown in Figure 1B, after selection in puromycin, the Id-1 stable transfectants showed constitutively high levels of Id-1 protein expression compared to the vector controls when cultured in serum-free conditions.

The article "Id-1 stimulates cell proliferation through activation of EGFR in ovarian cancer cells" was retracted in 2021. Reasons: duplicated images; concerns about the data.

### Effect of Id-1 expression on serum-independent cell proliferation in ovarian cancer cells

To investigate the effect of Id-1 expression on ovarian cancer cell proliferation, the DNA synthesis rate and the cell cycle S-phase fraction were determined using BrdU staining and cell cycle analysis, respectively, in the cells cultured in SFM. As shown in Figure 2

**Figure 2:** Effect of ectopic Id-1 expression on ovarian cancer cell proliferation. (**A**) BrdU incorporation rate between the Id-1 transfectants and the vector controls. Cells were cultured in SFM for 48 and 72 h, respectively, and stained with an antibody against BrdU. At least 500 cells were counted in each experiment and the percentage of BrdU-positive cells was calculated and compared with the vector controls at 48 h time point, which was assigned as 1. Results presented as the mean and standard deviation from three experiments. (**B**) Representative results of BrdU staining. Strong nuclear FITC-positive signal was considered as BrdU positive. The background was enhanced to facilitate the counting of total cell numbers. Note that the percentage of BrdU-positive cells is higher in Id-1 transfectants than the pBabe control transfectants.

, after culturing in SFM for 48 and 72 h, the percentage of BrdU-positive cells in Id-1 transfectants (solid columns) was higher than the vector controls (open columns) in all three ovarian cancer cell lines, especially in Ovca432 (up to 10-fold increase). The small increase of BrdU incorporation in Ovca433 Id-1 transfectant (approximately 1.7–2-fold) may be due to the relatively high basal levels of Id-1 in the parental cells, which may facilitate cell proliferation in SFM conditions. Nevertheless, these results indicate that ectopic expression of Id-1 in ovarian cancer cells led to increased DNA synthesis rate. To confirm these results, we performed flow cytometric analysis and studied the S-phase fraction. As shown in Figure 3

**Figure 3:** Effect of ectopic Id-1 expression on cell cycle S-phase fraction. Flow cytometric analysis was performed on the Id-1 and pBabe transfectants after culturing in SFM for 48 and 72 h, respectively. Note that the percentage of S cells is higher in Id-1 transfectants than in the vector control.

, the Id-1 transfectants from all three cell lines showed higher percentage of S-phase cells after culturing in SFM for 48 and 72 h, respectively. For example, the S-phase fraction was 25.17% in Ovca432–Id-1 transfectant, while the vector control only had 9.72% of S-phase cells after culturing in SFM for 48 h. Taken together, these results suggest that upregulation of Id-1 promotes cell proliferation in ovarian cancer cells.

The article "Id-1 stimulates cell proliferation through activation of EGFR in ovarian cancer cells" was retracted in 2021. Reasons: duplicated images; concerns about the data.

### Effect of ectopic Id-1 expression on EGFR in ovarian cancer cells

As previously suggested, Id-1 promotes cell proliferation through EGFR pathway in prostate cancer cells (Ling *et al*, 2004). Next, we studied if the Id-1-induced cell proliferation in ovarian cancer cells was mediated through EGFR pathway. As shown in Figure 4A

**Figure 4:** Effect of ectopic Id-1 expression on EGFR. (**A**) EGFR protein expression in the Id-1 transfectants and the vector control cells were cultured in SFM for 48 h and EGFR expression was examined by Western blotting. (**B**) EGFR promoter activity in Ovca420, Ovca432 and Ovca433 cells transiently transfected with pcDNAId-1 and the vector control pcDNA. pER-1 (luciferase reporter containing the EGFR promoter) and pRL-CMV-Luc (internal control) was cotransfected with pcDNA or pcDNA-Id-1, respectively. Cells were lysed 48 h after transfection and assayed for luciferase activity using the Dual-luciferase reporter assay system (Promega, WI, USA). The luciferase activity of the cells transfected with pER-1 and pcDNA was considered as 100%. Each experiment was repeated three times and the error bars represent the standard deviation from three independent experiments. Note that ectopic expression of Id-1 in Ovca420, Ovca432 and Ovca433 cells induces upregulation of EGFR at both transcriptional and protein levels.

, the vector-transfected control Ovca420 and Ovca433 cells showed detectable basal levels of EGFR protein, while EGFR was absent in Ovca432 cells. After exogenous Id-1 expression, the EGFR protein level was increased remarkably in all of the Id-1 transfectants compared with the vector control, suggesting that ectopic Id-1 expression resulted in upregulation of EGFR protein expression.

To confirm these results, luciferase assay was performed to examine if ectopic Id-1 expression could lead to EGFR activation at transcriptional level. After cotransfection of pcDNA-Id-1 or pcDNA vectors with pER-1 (luciferase reporter containing the EGFR promoter) and pRL-CMV-Luc (internal control) in the parental cell lines, we found that the EGFR promoter activity was increased in all three cell lines transfected with the Id-1 expression vector (solid columns, 250–350% increase) than the cells transfected with the pcDNA vector control (open columns) (Figure 4B). Taken together, these results indicate that upregulation of Id-1 in Ovca420, Ovca432 and Ovca433 cells has led to the upregulation of EGFR expression at both transcriptional and protein levels.

The article "Id-1 stimulates cell proliferation through activation of EGFR in ovarian cancer cells" was retracted in 2021. Reasons: duplicated images; concerns about the data.

### Effect of antisense Id-1 on the expression of EGFR in ovarian cancer cells

To further confirm the association between Id-1 and EGFR expression, we next studied whether blockage of Id-1 expression could lead to the downregulation of EGFR. As shown in Figure 1A, the Skov3 and Ovca429 cell lines had constitutively high levels of Id-1 expression regardless of serum concentrations; we then transfected a vector containing the antisense sequence to the Id-1 gene (Ling *et al*, 2003) into these two cell lines and tested the expression of EGFR. As shown in Figure 5A

**Figure 5:** Effect of Id-1 inactivation on EGFR. (**A**) Id-1 and EGFR protein expression in ovarian cancer cells transiently transfected with an antisense Id-1 expression vector (pcDNA-Id-1-AS) and the control vector (pcDNA). Cells were cultured in SFM for 48 h after transfection and Id-1 and EGFR expression was examined by Western blotting. (**B**) EGFR promoter activity in ovarian cancer cells transiently transfected with Id1-AS and the vector control. pER-1 (luciferase reporter containing the EGFR promoter) and pRL-CMV-Luc (internal control) were cotransfected with pcDNA or pcDNA-Id-1-AS, respectively, to Skov3 and Ovca429 cells. Cells were lysed for luciferase assays 48 h after transfection and the luciferase activity was tested using the Dual-luciferase reporter assay system (Promega, WI, USA). Samples transfected with pER-1 and pcDNA was considered as 100%. The error bars represent standard deviation from three independent experiments. Note that inhibition of Id-1 expression in Skov3 and Ovca429 cells reduces EGFR expression at both transcriptional and protein levels.

, 48 h after transfection, the Id-1 protein level was decreased in both cell lines compared to the pcDNA vector control (up to 70% decrease), indicating a successful inhibition of Id-1 expression in these cells. In addition, the expression of the EGFR protein was also downregulated at similar levels in these two cell lines. For example, Id-1 expression was decreased by 70% in Skov3 cells and the EGFR protein level was also reduced by approximately 70% compared to the vector-transfected cells. These results were further confirmed by luciferase assay, which showed that the EGFR promoter activity was inhibited in the cells transfected with the antisense Id-1 vector (solid columns) compared to the vector control (open columns) (Figure 5B). These results further support the hypothesis that Id-1 may be an upstream regulator of the EGFR signalling pathway.

The article "Id-1 stimulates cell proliferation through activation of EGFR in ovarian cancer cells" was retracted in 2021. Reasons: duplicated images; concerns about the data.

## DISCUSSION

In this study, we have demonstrated the positive effect of Id-1 expression on cell proliferation in three ovarian cancer cell lines (Figures 1, 2, and 3). In addition, the evidence provided in this study that ectopic expression (or downregulation) of Id-1 led to upregulation (or downregulation) of EGFR at both transcriptional and protein levels indicates that Id-1 may be an upstream positive regulator of the EGFR signalling pathway (Figures 4 and 5). Since upregulation of EGFR is a common event in ovarian cancer, our evidence implicates a novel mechanism responsible for EGFR activation in this cancer. As EGFR is one of the key factors in promoting ovarian cancer cell growth (Alper *et al*, 2000, 2001; Pack *et al*, 2004), our results also suggest an alternative target to suppress EGFR signalling pathway through inactivation of Id-1, thus inhibiting cancer cell growth. Although the Id-1-induced cell proliferation in normal as well as in cancer cells has been reported in several previous studies (Lin *et al*, 2000; Ouyang *et al*, 2002b; Wang *et al*, 2002b), this study is the first to demonstrate its positive role on ovarian cancer cell growth, especially its relation with EGFR pathway in ovarian cancer cells.

Several mechanisms have been suggested for the role of Id-1 in cell proliferation. For example, Id-1 inhibits p16^INK4a^/RB pathway leading to the bypass of replicative senescence in primary cells (Alani *et al*, 2001; Ohtani *et al*, 2001) and induces serum-independent proliferation in human prostate cancer cells (Ouyang *et al*, 2002b). Recently, the Id-1-induced cell proliferation has been linked to the Raf-MEK and NF-*κ*B pathways (Ohtani *et al*, 2001; Ling *et al*, 2002, 2003). Since Id-1 is a regulator of transcription, it is not surprising that it may regulate gene expression involving multiple signalling pathways. In this study, we found that ectopic Id-1 expression led to transcriptional activation of EGFR (Figure 4), while inactivation of Id-1 resulted in suppression of EGFR expression (Figure 5). Our results indicate a novel downstream effector of Id-1 in ovarian cancer cells. It is possible that increased Id-1 expression in ovarian cancer cells may provide autocrine signals to stimulate EGFR activity, resulting in promotion of cell proliferation. Since inactivation of EGFR has shown promising results in inhibition of ovarian cancer cell growth as well as suppression of metastatic phenotypes, our results suggest a new target in inhibition of EGFR signalling. Previously, it was also reported that Id-1 protected against anticancer drug taxol-induced cell death in nasopharyngeal carcinoma cells (Cheung *et al*, 2004) and suppression of Id-1 resulted in sensitisation to TNF*α*-induced apoptosis in prostate cancer cells (Ling *et al*, 2003). Since the front-line treatment strategy for advanced ovarian cancers is chemotherapy, downregulation of Id-1 may provide a novel strategy in improving the efficiency of chemotherapeutic drugs through suppression of Id-1-induced protection against apoptosis.

The article "Id-1 stimulates cell proliferation through activation of EGFR in ovarian cancer cells" was retracted in 2021. Reasons: duplicated images; concerns about the data.

Activation of EGFR as well as upregulation of Id-1 have been associated with aggressive behaviour and poor clinical outcome in ovarian cancer patients, respectively (Schindl *et al*, 2003; Skirnisdottir *et al*, 2004). In this study, we also found that the cell lines (i.e. Ovca432, Ovca433) that showed serum-dependent Id-1 expression had lower basal levels of EGFR and exhibited less invasive characteristics as reported in previous studies than the ones with serum-independent Id-1 expression (i.e. Ovca429) (Ellerbroek *et al*, 1998; Ahmed *et al*, 2002). These results further suggest a strong link between Id-1 and EGFR in promoting ovarian cancer progression. Recently, the positive role of Id-1 in metastasis has been reported through promoting tumour angiogenesis in a breast cancer animal model (Fong *et al*, 2003). In ovarian cancer, similar effects have been reported in the cells expressing high levels of EGFR. For example, Ovca8 cells expressing high levels of EGFR were much more invasive and contained high levels of integrins and MMP activity and these malignant phenotypes were suppressed when EGFR was inactivated through antisense technology (Alper *et al*, 2001). It is possible that increased expression of Id-1 and EGFR proteins may provide growth advantage for ovarian cancer cells to progress to more advanced malignant phenotype leading to poor prognosis in patients. However, how Id-1 and EGFR interact with each other and what signalling pathways are responsible for mediating ovarian cancer proliferation and progression remain to be elucidated.

In summary, we have provided first evidence that Id-1 plays an important part in the proliferation of ovarian cancer cells and this function is mediated through upregulation of EGFR. Although further investigations are needed to elucidate the precise molecular mechanisms responsible for the role of Id-1 in ovarian cancer, our results suggest a novel upstream regulator of the EGFR pathway. Since inhibition of EGFR is effective in the suppression of ovarian cancer cell growth, inactivation of Id-1 may provide an alternative strategy for the treatment of this cancer.
